# Novel Insights Into the Role of Mitochondria-Derived Peptides in Myocardial Infarction

**DOI:** 10.3389/fphys.2021.750177

**Published:** 2021-10-28

**Authors:** Dan Wu, Enny Kampmann, Geng Qian

**Affiliations:** ^1^Department of Cardiology, The First Medical Center, Chinese People’s Liberation Army Hospital, Medical School of Chinese People’s Liberation Army, Beijing, China; ^2^School of Life Sciences, City College of San Francisco, San Francisco, CA, United States

**Keywords:** myocardial infarction, mitochondria-derived peptides, mitochondria, mitochondria-ER communication, heart

## Abstract

Mitochondria-derived peptides (MDPs) are a new class of bioactive peptides encoded by small open reading frames (sORFs) within known mitochondrial DNA (mtDNA) genes. MDPs may affect the expression of nuclear genes and play cytoprotective roles against chronic and age-related diseases by maintaining mitochondrial function and cell viability in the face of metabolic stress and cytotoxic insults. In this review, we summarize clinical and experimental findings indicating that MDPs act as local and systemic regulators of glucose homeostasis, immune and inflammatory responses, mitochondrial function, and adaptive stress responses, and focus on evidence supporting the protective effects of MDPs against myocardial infarction. These insights into MDPs actions suggest their potential in the treatment of cardiovascular diseases and should encourage further research in this field.

## Introduction

Mitochondria are semi-autonomous, double-membrane organelles that play critical roles in maintaining cellular homeostasis by governing cell energy metabolism and influencing signal transduction, reactive oxygen species (ROS)-mediated oxidative stress, and apoptosis (Brooks, 2018; Cao et al., 2020). Mitochondrial biogenesis is a highly dynamic process, and the rapid recycling and turnover of mitochondrial components enables these organelles to adapt to metabolic changes resulting from different cellular stressors (Del Campo, 2019; Chiang et al., 2020; Jin et al., 2021). Thus, a decline in mitochondrial function is frequently associated with numerous diseases. Extensive research sought to elucidate how mitochondria dysfunction affects the onset and progression of myocardial infarction (MI), a condition characterized by impaired ATP synthesis and energy metabolism, enhanced apoptosis, and abnormal Ca^2+^ dynamics in cardiac cells (Sommer et al., 2016; Daiber and Münzel, 2020; Fender et al., 2020; Gori et al., 2020).

Cellular homeostasis is critically regulated by the interaction between mitochondria and the cell nucleus via coordinated expression of mitochondrial and nuclear genes. Importantly, this genetic crosstalk also allows cells to cope with environmental and metabolic stress (Ryan and Hoogenraad, 2007; Quirós et al., 2016). The mitochondrial DNA (mtDNA) contains 37 genes that encode 13 polypeptides, all subunits of the electron transport chain (ETC) (Mangalhara and Shadel, 2018), as well as 2 ribosomal RNAs (rRNAs) and 22 transfer RNAs (tRNAs) that are required for their translation (Michel et al., 2015). In contrast with nuclear-encoded genes, the synthesis of mitochondrial proteins is independent of the translational machinery associated with the endoplasmic reticulum. Still, mtDNA-encoded proteins represent only ∼1% of the mitochondrial proteome, which is estimated at up to 1,500 proteins that are therefore predominantly encoded by nuclear DNA (Calvo and Mootha, 2010).

Mitochondria-derived peptides (MDPs) conform a new class of peptides encoded by small open reading frames (sORFs) within known mtDNA genes (Yen et al., 2013; Kim et al., 2017). MDPs are widely distributed in various tissues such as heart, vascular wall, kidney, skeletal muscle, and colon. MDPs were shown to affect the expression of nuclear genes and play cytoprotective roles through maintaining mitochondrial function and cell viability under both normal and pathological conditions (Krejcova et al., 2004; Tajima et al., 2005). In this review, we summarize the effects of MDPs on immune and inflammatory responses, glucose homeostasis, mitochondrial function, adaptive stress responses, and apoptosis, and discuss the protective actions of MDPs against MI (Mottis et al., 2019). We hope this information will stimulate further research to materialize the therapeutic potential of MDPs in the treatment of MI and cardiovascular disease.

## Classification and Functions of Mitochondria-Derived Peptides

Eight MDPs have been identified up to date, all of them transcribed from sORFs harbored in mtDNA genes encoding 12S rRNA and 16S rRNA transcripts (Lee et al., 2015). The 12S rRNA gene is 954 nucleotides long, extends from nucleotides 648 to 1,601 (representing about 6% of the full mtDNA), and the encoded product presents a conserved secondary structure. The 16S rRNA gene is 1,559 nucleotides long and extends between nucleotides 1,671–3,229 of the mtDNA (Galtier et al., 2006). Several studies confirmed that MDPs regulate cellular metabolism and survival by maintaining glucose homeostasis, antioxidant capacity, and antiapoptotic signaling by binding to intracellular and extracellular receptors through autocrine and paracrine mechanisms (Yang et al., 2019).

### Humanin

Humanin (HN), the first discovered MDP, was identified in the brain of a patient with Alzheimer’s disease (AD) by Hashimoto and his team in 2001 (Hashimoto et al., 2001). Through different translational machineries, two HN peptides, 21 and 24 amino acids long, are produced, respectively, in mitochondrial and cytoplasmic compartments from a sORF located in the 16S rRNA gene of mtDNA (Sreekumar and Kannan, 2020). HN is found in circulating body fluids, such as blood and cerebrospinal fluid, and in metabolically active organs such as the heart, liver, and kidneys (Arakawa et al., 2008; Muzumdar et al., 2009; Chin et al., 2013). In addition, nuclear DNA contains several ORF sites, highly homologous to the mtDNA sequence encoding HN, which potentially give rise to several HN-like peptides (Jiang et al., 2020; Jusic and Devaux, 2020).

Humanin and its synthetic analogs have been shown to have significant cytoprotective and glucose-lowering effects. For example, the HN analog S14G (HNG) produced by substitution of serine by glycine at position 14 in HN, is 1,000 times more potent than HN (Arakawa et al., 2008). In turn, the HN homolog HNGF6A, formed by an additional substitution of phenylalanine by alanine at position 6, was shown to have an even greater effect than HN and HNG in improving central insulin sensitivity and lowering blood glucose levels in diabetic rats by counteracting the proapoptotic actions of insulin like growth factor binding protein-3 (IGFBP-3) (Muzumdar et al., 2009). Indeed, extensive research demonstrated that HN plays a protective role against various pathological conditions, including neurodegenerative diseases (Cui et al., 2017), diabetes (Xie et al., 2014), endothelial dysfunction (Ding et al., 2019), and cardiovascular disease (Ren et al., 2020).

#### Apoptosis

The antiapoptotic action of HN has been shown to result from inhibition of Bax-induced pore formation in the mitochondrial outer membrane and subsequent suppression of cytochrome c release (Ma and Liu, 2018). Besides, HN was shown to engage the Bid BH3 domain, which mediates the association of Bid with other Bcl-2 family members (Choi et al., 2007), and to bind directly to the extra-long isoform of Bim (BimEL). The ensuing inhibition of BimEL may thus contribute to the antiapoptotic properties of HN (Luciano et al., 2005). The therapeutic potential of HN as an antiapoptotic agent has been confirmed by *in vitro* and *in vivo* experiments demonstrating increased neuroprotection after HN binding to IGFBP-3 (Lee et al., 2013).

#### Oxidative Stress

Recent research also unveiled significant antioxidant properties for HN and its derivatives. In cardiac myoblasts challenged with H_2_O_2_, exposure to HNG lowered ROS levels, preserved mitochondrial membrane potential and ATP levels, induced activation of catalase and glutathione peroxidase, and decreased the ratio of oxidized to reduced glutathione (GSH) (Klein et al., 2013). Along these lines, HNG showed to beneficially regulate GSH and sphingolipid metabolism in a rat model of diet-induced obesity [46].

#### Inflammation

Zhao et al. (2013) showed that pretreatment with HN decreased the secretion of proinflammatory cytokines, i.e., interleukin (IL)-6, IL-1β, and tumor necrosis factor α (TNFα), induced by lipopolysaccharide (LPS) in cultured astrocytes. In turn, Jung et al. (2020) reported that intravenously administered HN promoted a “reparative” microglia phenotype characterized by enhanced phagocytosis and reduced proinflammatory responses in a mouse model of intracerebral hemorrhage.

#### Regulation of Mitochondrial Function

Many studies have examined the role of HN in the regulation of mitochondrial homeostasis. Experiments in human retinal pigment epithelial cells showed that HN exposure preserved essential functions related to energy production by increasing basal oxygen consumption rate, maximum respiration rate, respiration capacity, and ATP production (Sreekumar et al., 2016; Kleinbongard, 2020; Lahiri et al., 2020; Lindner et al., 2020). In pancreatic MIN6 β-cells, HN promoted mitochondrial biogenesis by increasing mitochondrial mass, mtDNA copy number, and PGC-1α, NRF1, and mitochondrial transcription factor A (mtTFA) levels (Qin et al., 2018b). Similarly, the HN analog HNG counteracted oxidative stress-induced mitochondrial dysfunction in cardiac tissue by reducing ROS generation and stabilizing mitochondrial membrane potential, mitochondrial structure, and ATP levels (Klein et al., 2013; Lobo-Gonzalez et al., 2020; Lyu et al., 2020; Sawashita et al., 2020). However, further research is needed to clarify the specific mechanisms by which HN sustains mitochondrial integrity and function in mammalian cells.

### MOTS-c

Mitochondrial open reading frame of the 12S rRNA-c (MOTS-c) is a 16-amino-acid peptide encoded by a sORF within the mitochondrial 12S rRNA. Originally identified by Lee et al. (2015) in various tissues in rodents, as well as in human plasma, MOTS-c proved to be an effective regulator of insulin sensitivity and metabolic homeostasis by inducing activation of AMP-activated protein kinase (AMPK). Subsequently, Kim et al. showed that MOTS-c can translocate to the nucleus in response to metabolic or oxidative stress, suggesting a novel role for MOTS-c in gene expression regulation via retrograde (mitochondria to nucleus) signaling (Quirós et al., 2016). Additional reports in animal models pointed out that MOTS-c regulates insulin resistance and attenuates the symptoms of hyperinsulinemia, obesity, and osteoporosis (Lee et al., 2015, 2016; Ming et al., 2016; Hu and Chen, 2018; Qin et al., 2018a; Lu et al., 2019; Mehta et al., 2019; Yan et al., 2019; Weng et al., 2021). Moreover, MOTS-c was shown to possess significant anti-inflammatory actions by inhibiting the expression of immune-related genes (Zhai et al., 2017; Li et al., 2018; Yan et al., 2019). Recently, Jiang et al. (2021) reported that MOTS-c administration enhanced object and location recognition memory formation and consolidation in mice treated with amyloid-beta peptide (Aβ1-42) or LPS through activation of hippocampal AMPK.

### Small Humanin-Like Peptides (SHLPs)

Small humanin-like peptides (SHLP1-6) are encoded and translated from a sORF contained within the same 16S RNA gene harboring the HN-encoding sORF (Cobb et al., 2016). Fist identified by Cobb et al. (2016), the 20–38 amino-acid-long SHLP peptides were shown to be expressed in mouse tissues including heart, liver, brain, kidney, spleen, prostate, testis, and skeletal muscle. Using RT-PCR, a mitochondrial origin was established for SHLPs 1, 4, 5, and 6, whereas SHLP2 and SHLP3 were amplified from both mitochondrial and nuclear cDNA (Cobb et al., 2016). These authors also found that circulating SHLP2 levels decline with age, and that male mice had higher SHLP2 levels than female mice in both the young and old groups. These results indicated that SHLP2 secretion levels vary with age and sex.

The Cobb et al. (2016) study showed that similar to HN, the neuroprotective actions of SHLP2 were associated with phosphorylation of both extracellular signal-regulated kinase (ERK) and signal transducer and activator of transcription 3 (STAT-3). Concordant also with HN effects, both SHLP2 and SHLP3 were shown to improve mitochondrial quality control, enhance oxidant consumption rate, mitochondrial biogenesis, and ATP synthesis, and mediate anti-apoptotic effects (Cobb et al., 2016). The beneficial influence of SHLP2 and SHLP3 on age-related neurodegenerative disease is supported by evidence that both SHLP2 and SHLP3 improved neuronal survival following toxic insults (Cobb et al., 2016). In particular, a prominent antiapoptotic effect was revealed for SHLP2 both in neurons treated with Aβ1-42 (Cobb et al., 2016) and in age-related macular degeneration (AMD) cybrid cells containing mtDNA from AMD patients [REF]. Several studies reported additional roles for SHLPs in the modulation of cardiovascular function, insulin sensitization, inflammation, and GSH and sphingolipid metabolism [46]. Interestingly, low circulating levels of SHLP2 were linked with increased risk of prostate cancer (Xiao et al., 2017; Mehta et al., 2019). Although these findings consistently affirm the beneficial actions of SHLPs on human health, further work is needed to elucidate the specific mechanisms mediating SHLPs’ effects.

## Protective Actions of Mitochondria-Derived Peptides Against Risk Factors for Myocardial Infarction

Ischemic heart disease is the leading cause of morbidity and mortality in the world (Reed et al., 2017; Qiao et al., 2021; Wischmann et al., 2020; Yang Y. et al., 2020; Zhang L. et al., 2020). It develops as a consequence of risk factors such as systemic arterial hypertension, left ventricular (LV) hypertrophy, hyperlipidemia, atherosclerosis, insulin resistance, diabetes, and aging (Ollauri-Ibáñez et al., 2020; Wang et al., 2020e; Watson et al., 2020; Winter et al., 2020). Indeed, age represents the largest risk factor for cardiovascular diseases, including cardiac fibrosis, atrial fibrillation, and heart failure (Steenman and Lande, 2017; Santosa et al., 2020; Schinner et al., 2020; Seano and Jain, 2020; Selvaraju et al., 2020). As mentioned, a correlation between MDP expression and age-related diseases is suggested by the significant decline in circulating MDP levels that occurs with age (Cobb et al., 2016). Since oxidative stress and mitochondrial dysfunction are tightly involved in the mechanisms of age-related diseases, MDPs, especially HN and MOTS-c, the most studied ones, have emerged as promising therapeutic targets to treat neurological, cardiovascular, and metabolic conditions associated with advanced age (Zapała et al., 2010; Thummasorn et al., 2017; Yang et al., 2019; Kim et al., 2021).

Mitochondria-derived peptides were shown to critically influence lipid and glucose metabolism, two aspects closely related with myocardial disfunction and infarction. Cobb et al. (2016) reported that SHLP2 and SHLP3 enhanced 3T3-L1 pre-adipocyte differentiation and increased leptin levels in mice. Meanwhile increased peripheral glucose uptake and suppressed hepatic glucose production were observed after intracerebral infusion of SHLP2 in rats subjected to systemic pancreatic insulin clamp and physiologic hyperinsulinemic-euglycemic clamp (Cobb et al., 2016). This suggests that central activity of SHLP2 has obvious peripheral effects. Gong et al. (2015) showed that intraperitoneal administration of the HN homolog HNG can reduce weight, visceral fat contents, and hepatic steatosis in high-fat diet (HFD)-fed mice. It is unclear, however, whether reduced adipogenesis or increased lipolysis mediated these effects. Lee et al. reported that MOTS-c enhanced lipid oxidation and glucose metabolism in skeletal muscle by increasing the expression of GLUT4 and inhibiting the folate-methionine cycle. The ensuing inhibition of *de novo* purine synthesis caused accumulation of endogenous 5-aminoimidazole-4-carboxamide ribonucleoside (AICAR), a purine precursor, leading to activation of AMPK. Because *de novo* purine synthesis is subjected to feedback regulation by purine nucleotides, MOTS-c was proposed to accelerate *de novo* purine synthesis, which is consistent with the observed increase in NAD^+^ levels, glycolytic fluxes, and increased routing of glucose to the pentose phosphate pathway (PPP). Following AICAR accumulation, AMPK activation stimulates fatty acid oxidation via phosphorylation-induced inactivation of acetyl-CoA carboxylase (ACC) (Steinberg and Kemp, 2009). Studies from Lee et al. (2015) also showed that compared with control cells, HEK293 cells stably overexpressing MOTS-c exhibited higher levels of carnitine shuttles, reduced essential fatty acid levels, and increased levels of the β-oxidation intermediate myristoyl-CoA. These studies concluded that MOTS-c treatment prevented age-dependent and HFD-induced insulin resistance by enhancing GLUT4 expression and the rate of insulin-induced glucose utilization in skeletal muscle, without changes in the hepatic glucose production rate (Lee et al., 2015). In turn, Muzumdar et al. (2009) reported that intracerebroventricular administration of HN during pancreatic-euglycemic clamp increased insulin sensitivity, leading to a reduction in hepatic glucose production by inducing fatty acid metabolism and Akt signaling. Along these lines, Kuliawat et al. (2013) showed that glucose-stimulated insulin secretion was potently stimulated by the HN analog HNGF6A both in βTC3 cells and in pancreatic islets from normal and diabetic mice.

Coronary artery atherosclerosis, characterized by lipid deposition, foam cell formation, and accumulation of cholesterol in the arterial wall, is the leading cause of myocardial ischemia and coronary artery disease (Tabas et al., 2007; Lyu et al., 2015; Sawashita et al., 2020; Zhang Y. et al., 2020; Zhao et al., 2020). Excessive production of ROS, caused by long-term occlusion of the coronary artery, enhances oxidative stress and inflammation, resulting in vascular endothelial dysfunction and accelerated formation of atherosclerotic plaques (Lu et al., 2020; Watanabe et al., 2020; Wincewicz and Woltanowski, 2020; Yang Q.K. et al., 2020). The expression of HN in the endothelial cell layer of human arteries and veins was first reported by Bachar and colleagues. They showed, through *in vitro* experiments, that HN protected against atherosclerosis by reducing ROS production and attenuating oxidative stress (Bachar et al., 2010). The formation of foam cells results from imbalanced cholesterol influx and efflux in arterial wall-associated macrophages and contributes to the onset and development of atherosclerosis. Using cultured RAW 264.7 macrophages, Zhu et al. showed that HNG prevents ox-LDL-induced foam cell formation. This effect resulted from inhibition of CD36 and low-density lipoprotein receptor (LOX)-1 upregulation, which reduced ox-LDL endocytosis, coupled with upregulation of ATP-binding cassette (ABC) transporter A1 and ABCG1 levels, which enhanced ox-LDL efflux (Zhu et al., 2017). Hyperglycemia is an important contributor to the pathological development of atherosclerosis in diabetic patients. Wang et al. reported that HN treatment prevented high glucose-induced attachment of monocytes to human umbilical vein endothelial cells (HUVECs). This effect was mediated by ERK5 phosphorylation and induction of Krüppel-like factor 2 (KLF2) expression, upregulation of KLF2 target genes such as endothelial nitric oxide synthase (eNOs) and endothelin-1 (ET-1), and reduced expression of leukocyte adhesion molecules (VCAM-1 and E-selectin) (Wang et al., 2018). Qin et al. found that circulating MOTS-c levels were downregulated in patients with coronary endothelial dysfunction. They showed that plasma MOTS-c levels were positively correlated with microvascular and epicardial coronary endothelial function in study subjects, demonstrating also that exposure to MOTS-c had no direct vasoactive effects but improved acetylcholine-induced vasodilation in aortic explants from renal artery stenosis mice (Qin et al., 2018a).

### Role of Mitochondria-Derived Peptides in Myocardial Ischemic Injury and Ischemia/Reperfusion Injury

A pivotal feature of ischemia is the inadequate supply of oxygen to the mitochondria to support oxidative phosphorylation (OXPHOS). This causes excessive ROS production and oxidative stress injury, leading to myocardial cell death (Zhu et al., 2018; Zhou et al., 2019; Hughes et al., 2020; Wang et al., 2020c). Myocardial ischemic injury usually results in infarction, arrhythmias, and decreased myocardial contractility. Reperfusion therapy refers to procedures that allow the rapid return of blood flow to the ischemic area of the myocardium, through which mortality can be approximately halved (Jin et al., 2018; Smadja et al., 2020; Tan et al., 2020; Zhu et al., 2021). However, reperfusion itself may induce irreversible cell injury (e.g., necrosis and apoptosis), thus leading to extensive infarct size, diminished cardiac contractile function, and arrhythmia (Zhou et al., 2017a,b, 2018c; Szulcek et al., 2020; Wang et al., 2020d). The ensuing reconstruction of the damaged myocardium poses a big clinical challenge, as it is a key contributor to cardiac dysfunction after MI (Zhou et al., 2018b, 2020; Singh et al., 2020; Wang et al., 2020a). Myocardial fibrosis represents a secondary response to the pathophysiologic remodeling process. It involves profound changes in the interstitial myocardial collagen network, facilitating the development of cardiac dysfunction and arrhythmias and influencing the clinical course and outcome of heart failure patients (Zhou et al., 2018a; Tomita et al., 2020; Wang et al., 2020b).

Myocardial injury begins after about 20 min of coronary occlusion, first affecting the subendocardium and papillary muscle, and extending thereafter into the mid-myocardial bed-at-risk by about 60–90 min (Reimer et al., 1977). Myocardial injury may be reversible because of the activation of physiologic adaptations manifested in myocardial stunning, hibernation, and pre- and post-ischemic conditioning (Heyndrickx et al., 1975). However, prolonged ischemia causes irreversible myocardial injury regardless of the tissue’s hypoxic tolerance and intrinsic adaptive mechanisms. In this setting, oxygen consumption by oxidative phosphorylation and the synthesis of high energy phosphate products are reduced, along with decreased availability of malate (a complex I substrate) and succinate (a complex II substrate) in mitochondria (McCully et al., 2007). Alterations in complex I activity and accumulation of succinate during ischemia may be related to mitochondrial oxidative injury during reperfusion (Pacher et al., 2006). Here, the maximal rate of hydrolyzed succinate overwhelms the speed of ATP synthesis, leading to a phenomenon called reverse electron transport (RET) that results in enhanced ROS production by complex I. Accordingly, pharmacological inhibition of complex I slows the reactivation of mitochondria and reduces ROS (Chouchani et al., 2013). Multiple biochemical and ultrastructural changes occur in cardiac cells upon ischemia-induced ATP depletion. Faced with oxygen deprivation, the heart switches from fatty acid oxidation to anaerobic glycolysis to sustain ATP production, leading to the accumulation of lactate and a decline in cellular pH (Walker et al., 2000; Khabbaz et al., 2001). Intracellular acidification stimulates the activity of the Na^+^/H^+^ exchanger, which enhances in turn Ca^2+^ influx by activating the Na^+^/Ca^2+^ exchanger as a way to remove excess Na^+^ into the extracellular space. This leads eventually to mitochondrial Ca^2+^ overload, which ultimately results in mitochondrial swelling, increased mitochondrial intermembrane distance, and deficient OXPHOS (Pagliaro and Penna, 2015).

As with myocardial ischemic injury, the extent of ischemia/reperfusion (I/R) injury varies based upon reversible events, onset of reperfusion arrhythmias, cardiac stunning, etc., which determine the eventual occurrence of lethal reperfusion injury (Hausenloy et al., 2016). Clinically, I/R injury is associated with the disruption of the microvasculature leading to the no-reflow phenomenon and activation of inflammatory reactions (Wang et al., 2020b). Over the last decades, abundant research focusing on lethal myocardial reperfusion injury reported the mechanisms involved in this process. These alterations include rapid normalization of pH, intracellular Ca^2+^ overload, and ROS generation, all of which aggravate mitochondrial dysfunction (Pan et al., 2013). A hallmark of the latter is the opening of the mitochondrial permeability transition pore (mPTP), which is thought to be the most noxious step during reperfusion injury, leading to activation of apoptotic and necrotic signaling pathways (Ruiz-Meana et al., 2009).

Several studies suggested that HN or its synthetic analogs might be effective to treat MI. Recently, Wijenayake et al. uncovered the cytoprotective role of a humanin homolog (TSE-humanin), expressed in freshwater turtles, against sustained hypoxia and oxidative damage (Wijenayake and Storey, 2021). In a rat model of myocardial I/R injury, Thummasorn et al. showed that endogenous HN levels were decreased at the end of cardiac I/R. Interestingly, intravenous injection of HNG 15 min before I/R (but not during I/R) significantly decreased arrhythmia incidence and infarct size, improved cardiac mitochondrial function, and attenuated cardiac dysfunction. The same group later showed that high- dose HNG (252 μg/kg) administration during the ischemic phase increased myocardial HN levels, reduced arrhythmia, myocardial infarction area, and mitochondrial dysfunction. These effects were associated with AKT signaling activation, inhibition of Bax translocation to the mitochondrial membrane, and apoptosis prevention (Thummasorn et al., 2017). Subsequently, using isolated cardiac mitochondria, the same group showed that HNG was more effective than cyclosporine A in decreasing oxidative stress and alleviated mitochondrial damage caused by H_2_O_2_ by decreasing complex I activity (Thummasorn et al., 2018). Similarly, Muzumdar et al. showed that administration of HNG one hour before or at the time of reperfusion improved LV function and decreased infarct size in a mouse model of I/R. The suggested mechanism involved AMPK/eNOS signaling and downregulation of pro-apoptotic factors (Muzumdar et al., 2010).

### Role of Mitochondria-Derived Peptides in Post-infarction Cardiac Fibrosis

The development of post-MI heart failure is associated with complex and progressive cellular and ultrastructural transformation events resulting in ventricular remodeling, a phenomenon first described by Tennant and Wiggers in the 1930s (Tennant and Wiggers, 1935). The human left ventricle has 2 to 4 billion cardiomyocytes, and a MI can cause the death of ≥25% of this population in a few hours (Beltrami et al., 2001). Due to the heart’s limited ability for rapid self-repairing after catastrophic damage, scar formation, rather than muscle regeneration, is often the major component of the healing response following MI (Olivetti et al., 1991). The mechanisms of post-infarction cardiac remodeling include interactions between cellular, extracellular, and neurohormonal components. Early changes occurring within the first 72 h of an acute myocardial insult include expansion of the infarct zone, mainly because of the degradation of intermyocyte collagen struts by serine proteases and activated matrix metalloproteinases (MMPs) released from neutrophils. Concomitantly, myocardial necrosis determines an influx of inflammatory cells, including macrophages and other antigen-presenting cells, which results in wall thinning, ventricular dilatation, and eventually, cardiac rupture (Sutton and Sharpe, 2000). Late remodeling mainly involves eccentric hypertrophy and LV cavity dilation because of the increased load on the non-infarcted myocardium (Anversa et al., 1985). Adverse cardiac remodeling is facilitated by the imbalance between MMPs and their inhibitors (tissue inhibitors of metalloproteinases; TIMPs). These are regulated by several transcription factors and enzymes, including the NF-κB and JAK-STAT pathways, which are influenced by the renin-angiotensin-aldosterone system (RAAS) (Chen et al., 2004). Despite the extensive knowledge accumulated so far, clinical treatment of post-MI heart failure is still very challenging and thus requires further research.

Contrasting with the solid preclinical evidence supporting the beneficial actions of HN and its analogs in cardiac I/R injury, research on the possible influence of MDPs in cardiac remodeling remains scarce. Recently, Wei et al. (2020) reported that treatment with MOTS-c significantly decreased blood pressure, maintained normal cardiac structure, reversed ventricular remodeling, and reduced the stiffness of blood vessels in a rat model of vascular calcification induced by vitamin D3 plus nicotine (VDN) treatment. They further showed that MOTS-c attenuated VDN-induced vascular calcification pathology by stimulating AMPK signaling, reversing also the upregulation of angiotensin II type 1 (AT-1) and endothelin B (ET-B) receptors mediated by VDN. Overexpression of AT-1 receptors is linked to increased myocardial fibrosis and cardiac dysfunction, which is consistent with the beneficial effect of MOTS-c against both oxidative stress and development of myocardial contractile dysfunction (Honda et al., 2018). Regarding ET-B, experiments with the AMPK agonist AICAR indicated that AMPK activation downregulates ET-B receptor expression, stimulates autophagy, and normalizes contractile responses to the ET-B agonist sarafotoxin 6c in VSMCs cultured under high glucose conditions (Chen et al., 2018).

## Outlook and Perspectives

Mitochondrial dysfunction is closely correlated with the symptoms of MI and cardiovascular disease (Suárez-Rivero et al., 2016). Available data suggest that impaired synthesis of MDPs in cardiomyocytes and endothelial cells contributes to the pathological sequelae of cardiac I/R injury. Accordingly, treatment with MDPs was shown to alleviate ischemic injury, limit infarct area, and attenuate adverse cardiac remodeling after experimental infarction in rodent models. However, in the setting of MI, addressing the optimal time window at which MDPs exert maximal effects would help validate their use as pre-, per-, and/or post-conditioning agents. Collectively, the findings summarized above suggest the therapeutic potential of MDPs to treat MI as well as other common age-related diseases.

## Author Contributions

DW wrote the original manuscript. EK and GQ contributed to the manuscript revision. All authors approved the submission.

## Conflict of Interest

The authors declare that the research was conducted in the absence of any commercial or financial relationships that could be construed as a potential conflict of interest.

## Publisher’s Note

All claims expressed in this article are solely those of the authors and do not necessarily represent those of their affiliated organizations, or those of the publisher, the editors and the reviewers. Any product that may be evaluated in this article, or claim that may be made by its manufacturer, is not guaranteed or endorsed by the publisher.
